The article "Inducing apoptosis in acute myeloid leukemia; mechanisms and limitations" was published in 2024. Journal: Heliyon.

# Inducing apoptosis in acute myeloid leukemia; mechanisms and limitations

**DOI:** 10.1016/j.heliyon.2024.e41355

**Published:** 2024-12-19

**Authors:** Zahra Koolivand, Farbod Bahreini, Elham Rayzan, Nima Rezaei

**Affiliations:** a Faculty of Pharmacy and Pharmaceutical Sciences, Islamic Azad University, Tehran Medical Sciences University (IAUTMU), Tehran, Iran; b International Hematology/Oncology of Pediatrics Experts (IHOPE), Universal Scientific Education and Research Network (USERN), Tehran, Iran; c Department of Biochemistry, Faculty of Biological Sciences, Tarbiat Modares University, Tehran, Iran; d Network of Immunity in Infection, Malignancy and Autoimmunity (NIIMA), Universal Scientific Education and Research Network (USERN), Tehran, Iran; e Institute of Anatomy, University of Luebeck, Luebeck, Germany; f Research Center for Immunodeficiencies (RCID), Children's Medical Center, Tehran University of Medical Sciences, Tehran, Iran; g Department of Immunology, School of Medicine, Tehran University of Medical Sciences, Tehran, Iran

**Keywords:** Acute myeloid leukemia, BCL2 protein, Treatment failure, Multiple drug resistance, Apoptosis

## Abstract

Acute myeloid leukemia is the expansion of leukemic stem cells which might originate from a stem cell or a progenitor which has acquired self-renewal capacity. An aggregation of leukemic blasts in bone marrow, peripheral blood, and extramedullary tissue will result in acute myeloid leukemia. The main difficulty in treating acute myeloid leukemia is multidrug resistance, leading to treatment failure. This unfortunate phenomenon is practically elevated because of apoptosis inhibition in tumor cells.

Two general apoptotic pathways are the Bcl-2 regulated pathway (the intrinsic pathway) and the death receptor pathway. Deficiencies in each of these apoptotic pathways can cause the usual resistance mechanism in this disease. This article reviews and highlights different antiapoptotic pathways, currently-used treatments, and new findings in this field, which may lead to the development of treatment methods for acute myeloid leukemia.

## List of abbreviations

Acute myeloid leukemia: AML
complete remission: CR
inhibitor of apoptosis proteins: IAPs
murine double minute 2: MDM2
B cell lymphoma 2: BCL2
FMS-like tyrosine kinase 3: FLT3
internal tandem duplication: ITD
the tyrosine kinase domain: TKD
isocitrate dehydrogenase 1: IDH1
gemtuzumab ozogamicin: GO
natural killer: NK
tumor necrosis factor: TNF
TNF-related apoptosis-inducing ligand: TRAIL

## 1 Introduction

Acute myeloid leukemia (AML) is adults' most prevalent acute leukemia. It is a heterogeneous disease caused by irregular clonal proliferation of myeloid precursors, in which neutropenia, anemia, and thrombocytopenia may result from the disease. AML induces the accumulation of leukemic blasts in bone marrow, peripheral blood, and extramedullary tissue [1,2]. It should be considered that while differentiation of leukemic blasts is not entirely blocked in AML, several types of leukemic blasts can emerge from a single cell that does not differentiate at different stages of differentiation [3]. Each year, about 20,000 adults are diagnosed with AML in the United States. It is estimated that in 2023, more than 20,380 patients will be diagnosed with AML in the U.S., and the gender distribution is estimated to be near 11,410 (⁓55 %) in males and 8970 in females (⁓45 %). Among the diagnosed patients, it is evaluated that, unfortunately, nearly 11,310 deaths would be recorded, and it is estimated that the gender distribution would be 6440 for males (⁓56 %) and 4870 deaths in females (⁓44 %) [4]. According to the World Health Organization (WHO) classification, AML is classified into six major groups, including AML with recurrent genetic abnormalities, AML with myelodysplasia-related changes, AML with therapy-related myeloid neoplasms, AML that is not otherwise specified, Myeloid sarcoma and Myeloid proliferations related to Down syndrome [5]. Although several studies have been performed to detect genetic mutations responsible for AML pathogenesis, the treatment methods have not significantly changed in the past two decades as most genetic defects are still unknown [6]. Depending on whether the patients’ chromosomes have undergone modifications, the karyotypes of AML patients might be either normal or aberrant. Therefore, the primary variable used by physicians to assess the disease prognosis for AML is the karyotype. This is because the type and quantity of chromosomal abnormalities present in the karyotype could affect the severity of the disease [7]. Besides, due to the high possibility of relapse-related deaths in AML patients, the karyotype of leukemic cells is essential to predict complete remission (CR) and relapse rate [2].

Although 85 % of AML patients initially respond to chemotherapy, the duration of remission is short. CR and relapse are seen in about 80 % and 50 % of the cases after initial induction chemotherapy, respectively [8]. Unluckily, it has been demonstrated that in patients older than 70 years of age, the 3-year overall survival with induction chemotherapy is less than 20 %. Another common challenge in AML treatment is chemotherapy resistance, which will be described mechanistically in this review [9].

It is worth mentioning that deficiency in apoptotic pathways causes the usual mechanisms of disease and drug resistance, which promotes the survival of cancerous cells by inhibiting programmed cell death (so-called apoptosis) [10]. Cancers often exhibit a disrupted equilibrium between cell death and cell division, a phenomenon that can manifest during any phase of the apoptosis process [11]. Tumor development can be affected by various instabilities between proapoptotic and antiapoptotic molecules [12]. Identifying cellular pathways and genetic factors contributing to these mechanisms can result in recognizing possible prognostic biomarkers and treatment targets [13]. One pathway used by cancer cells to evade apoptosis is based on upregulated antiapoptotic BCL-2 proteins and TP53 gene mutation. Mutations in TP53 are observed in 5–10 % of de novo AML and 30–40 % of therapy-related cases and are considered important indicators of poor outcomes [14,15]. In non-complex karyotype AML cases, the TP53 locus is typically wild-type. However, missense mutations in TP53 are responsible for most changes and are frequently found in complex karyotypes, relapsed and elderly AML patients, and therapy-related AML. For cases without TP53 mutations, alternative mechanisms may obstruct apoptosis. Dysfunctional p53 is prevalent in AML due to changes in p53-regulatory proteins [[16], [17], [18], [19]]. In AML, TP53 gene expression may be more important than gene mutation, as nearly 90 % of AML patients show lowered expression levels [20,21]. Nearly 90 % of AML patients have exhibited the expression of the SMAC/DIABLO gene. Further, an elevated expression of this gene has been associated with higher rates of DFS and OS [22]. Pluta et al. have documented that SMAC/DIABLO protein levels are notably elevated in 98 % of AML patients and that this heightened expression serves as a reliable indication of extended OS and successful CR achievement [23].

Death receptor pathway and critical antiapoptotic factors that are effective in this regard are inhibitors of apoptosis proteins (IAPs), murine double minute 2 (MDM2), and antiapoptotic B cell lymphoma 2 (BCL2) proteins [24]. Targeting and identifying apoptosis pathways can play a pivotal role in treating cancers. Fig. 1 illustrates a brief schematic overview of the role of mutated p53 and overexpression of IAPs that play a role in AML cell survival and how available treatments like Embelin and Ventoclax (which will be discussed in this paper) can alter these mechanisms. Herein, this article strives to clarify different apoptosis pathways and reviews current drugs for treating AML.

**Fig. 1:** The molecular pathways involved in AML cell survival include the influences of upregulated anti-apoptotic proteins, overexpression of IAPs, and p53 mutations. These factors play a pivotal role in developing therapy resistance and relapse. Targeted therapies, such as Venetoclax and Embelin, are designed to interfere with these pathways by inhibiting anti-apoptotic proteins and IAPs, thereby enhancing the effectiveness of treatment.

## 2 Current methods in AML treatment

In the past years, a combination of cytarabine (Ara-c) and anthracycline has been used in induction therapy for patients who can tolerate intensive induction chemotherapy [25]. Anthracycline antibiotics such as idarubicin or daunorubicin and deoxycytidine analog (cytarabine) have been reported to be beneficial for CR in 50–75 % of cases [2]. Furthermore, in 2017, a liposomal formulation of cytarabine and daunorubicin at a 5:1 M ratio (CPX-351) was granted FDA approval for the treatment of newly diagnosed AML patients (CPX-351 (vyxeos) in AML. Furthermore, research indicates that azacitidine (HMA) provides a viable treatment alternative specifically tailored for elderly patients [26]. Results from clinical trials have manifested that the HMA can be used for maintenance therapy after induction therapy; they have also shown better survival with HMA compared to intensive treatment [9]. Nonetheless, the five-year survival rate of only 40 % of patients under 60 years of age is reported when these induction regimens have been employed [27].

FMS-like tyrosine kinase 3 (FLT3), which is only expressed in CD34^+^ hematopoietic stem cells, is a receptor tyrosine kinase. It has been involved in the apoptosis and differentiation of hematopoietic stem cells [28]. It is essential to note that hematopoietic stem cells, which typically progress through differentiation, can pause their division at various stages. This distinction, where cells halt division, serves as a key differentiation between carcinogenesis and leukemogenesis [29]. In almost 35 % of newly diagnosed AML patients, internal tandem duplication (ITD) in the transmembrane domain and Asp835Tyr mutation in the tyrosine kinase domain (TKD) of the FLT3 gene have been seen. It merits emphasis that these particular mutations are considered significantly relevant in the context of this study [30]. Indeed, FLT3-ITD represents the predominant manifestation of FLT3 mutation correlated with an elevated incidence of relapse and clinical outcomes, whereas FLT3-KTD mutations have not been conclusively linked to unfavorable prognosis [31,32]. In November 2018, Gilteritinib (XOSPATA) was granted FDA-approval for treatment of adult patients with relapsed or refractory AML with a FLT3 mutation [33]. Recently, In july 2023, another FLT3 inhibitor, Quizartinib (Vanflyta) was granted FDA approval to be used as a combination therapy with standard Cytarabine and Anthracycline induction and Cytarabine consolidation and as a maintenance monotherapy following consolidation chemotherapy, in adult patients with newly diagnosed AML with FLT3 internal tandem duplication (ITD)-positi [34]. In fact, Quizartinib, along with its primary active metabolite AC886, exhibits adequate affinity for the ATP binding domain of FLT3, and both manifest a ten-fold reduced affinity for the FLT3-ITD mutation relative to FLT3 in an ATP binding assay. The inhibitory action of Quizartinib and AC886 extends to the suppression of FLT3 kinase activity, thereby inhibiting receptor autophosphorylation and consequently suppressing the downstream FLT3 receptor signaling, thereby inhibiting cell growth dependent on FLT3-ITD [32,35]. In general, tyrosine kinases have a pivotal role in growth factor signaling modification and consequently play a significant role in various cellular regulatory processes [36]. It has been established that mutations in tyrosine kinase act as a catalyst for uncontrolled proliferation within cytokine-dependent cell lines [37]. Clinical trials on patients with FLT3 mutations have shown that adding a kinase inhibitor named midostaurin (a multitargeted kinase inhibitor) to their induction chemotherapy improved OS [38]. Midostaurin and its metabolites play their roles by only targeting mutant forms of FLT3 and have shown a desirable safety profile. However, in addition to Midostaurin, other FLT3 inhibitors, including Sorafenib, Lestaurtinib, Quizartinib, Gilteritinib, and Crenolanib, are in the stage of clinical studies [39].

Another crucial genetic abnormality in newly diagnosed AML patients is a mutation in isocitrate dehydrogenase 1 (IDH1) and IDH2, which encode enzymes effective in cellular metabolism. Therefore, Ivosidenib and Enasidenib were granted FDA approval to treat newly diagnosed AML patients by inhibiting the mutant forms of IDH proteins [40].

In 2017, gemtuzumab ozogamicin (GO), which is an antibody-drug conjugate, was granted FDA approval to be added to the induction chemotherapy for adult patients with newly diagnosed CD33^+^ AML. Notably, CD33 (an AML antigen) is a candidate in this regard because of its high expression in leukemic cells [41]. On the other hand, in patients older than 60 years of age with CD33^+^ AML, GO has been approved as monotherapy for treatment. In addition to the previously mentioned treatment methods, allogeneic hematopoietic stem cell transplantation has remained an essential method for AML treatment [42]. Among the most updated immunotherapeutic treatment options for AML, natural killer (NK) cell immunotherapy has been recently introduced to the field. As the anti-tumor properties of NK cells make them great candidates for AML immunotherapy, various clinical trials are in progress to assess their effect and safety [43].

## 3 Apoptosis and AML treatment

### 3.1 Role of apoptosis in cancer progression

Hematological malignancies exhibit dysregulated programmed cell death genes, promoting genetic instability and oncogene activation [36]. Apoptosis, intricately characterized as a form of programmed cell death, is intricately orchestrated by a specific group of enzymes known as cysteine proteases, more commonly referred to as caspases. These enzymes play a crucial role in the cellular lifecycle, meticulously initiating and executing the cell death process as a vital mechanism for maintaining tissue homeostasis and overall organism health [44]. It has been well understood that apoptosis dysregulation increases neoplastic transformation and plays a critical role in autoimmune diseases and neurodegenerative disorders [13]. Indeed, tumor invasiveness and irregularities in cell proliferation occur because of a lack of apoptotic control, which allows cancer cells to survive longer [45].

Proteolytic enzymes called caspases (cysteine-aspartic proteases) are well known for regulating inflammation and cell death. Nevertheless, growing evidence shows that caspases have multiple uses in addition to apoptosis-like proliferation, tumor suppression, and neural development [46].

Generally, four pathways initiate caspase activation: 1- straight caspase activation, 2- pathway connected to the endoplasmic reticulum, 3- the mitochondrial pathway, and 4- death receptor pathway [47].

Two main apoptotic pathways are as follows: 1- the mitochondria-mediated apoptosis (intrinsic apoptosis pathway, BCL2 regulated pathway) that is dependent on the release of cytochrome C into the cytosol, and 2- the death receptor pathway (extrinsic pathway) [48]. Despite distinct initiation mechanisms, both pathways result in a common outcome: the activation of a series of proteolytic enzymes belonging to the caspase family [49]. In addition, some factors, such as deprivation of growth factor, viral infection, and DNA damage, activate the innate or BCL2-regulated pathway, which is controlled strictly by the Bcl2 family of proteins [50].

### 3.2 The antiapoptotic role of BCL2

The BCL2 family plays a critical role in apoptosis arrangements by regulating the intrinsic apoptosis pathway [12,51]. Certain types of AML may have issues with apoptosis. AML1-ETO fusion protein found in AML with t ([8,21]) can trigger BCL-2 transcription. The transcription factor CCAAT/enhancer binding protein α, encoded by the CEBPA gene, is mutated in approximately 10 % of AML patients and may induce BCL-2 expression [18,52]. As illustrated in Fig. 2, the formation of the Apaf1-cytochrome C complex is essential for the activation of caspase9. However, the mitochondrial release of cytochrome C can be prevented by BCL2 proteins, which ultimately inhibit apoptosis [53]. Promoting apoptosis can occur because of interactions between BH3-only proteins (which promote apoptosis and serve as death chaperons) and the BCL2 family [50]. On the other hand, compelling evidence has demonstrated that the downregulated levels of *Bcl2* mRNA can suppress cell apoptosis and increase cell proliferation in AML patients [54]. These studies reveal the double-edged sword effect of BCL2 proteins in AML. Nonetheless, the categorization of BCL2 proteins can be beneficial to manifest the effect of these proteins in AML.

**Fig. 2:** The intrinsic apoptosis pathway occurs when the cytochrome C-Apaf-1 complex activates caspase-9. This complex is formed only when mitochondria release cytochrome C. In general, the antiapoptotic proteins of the Bcl-2 family prevent apoptosis by stopping cytochrome C release from mitochondria. Venetoclax, Oblimersen, and Navitoclax can inhibit Bcl-2, which can lead to apoptosis. Obatoclax induces apoptosis by increasing the release of cytochrome C from mitochondria. The extrinsic and intrinsic apoptosis pathways can be connected through tBID. TRAILR2, TRAILR1 receptors, and Fas bind to their intrinsic ligands and form the death-inducing signaling complex (DISC) which ultimately leads to caspase-8 activation and initiates cell apoptosis. Ultimately, Caspase-8 activation leads to the cleavage of BID. Activation of Caspase-9 and Caspase-8 from both apoptosis pathways ultimately results in the activation of Caspase-3 and Caspase-7, leading to apoptosis.

In this regard, the BCL2 family can be subsumed into three main categories.

1) Those which inhibit apoptosis, consist of BCL2L1, MCL1, BCL2, BCLW, A1, and BCLB [50]. It has been demonstrated that BCL2L1 plays a vital role in hematological malignancies and participates in drug resistance mechanisms. BCL2L1 has also been shown to be essential for embryogenesis and plays a significant role in the survival of platelets. It is worth mentioning that thrombocytopenia and lymphopenia can be developed by BCL2L1 and BCL2 antagonisms [55]. Moreover, the life span of mature B and T lymphocytes depends on BCL2 (i.e., BCL2 positively affects the life span of these lymphocytes) [56]. MCL1 has been involved in resistance to BCL2 inhibitors in cancer therapy [57]. Hence, MCL1 is necessary for the survival of progenitor T and B lymphocytes and hematopoietic stem cells [56].
2) Those which increase apoptosis consist of BAK, BOK, and BAX [50]. MCL1 applies its function by antagonizing BAK and BAX activation, which supports the bioenergetic function of mitochondria and facilitates its homeostasis [58].

These first two categories have four BH domains (BH 1–4) [59]. It should be considered that this category is activated adversely from the first category [53]. In essence, BAK and BAX are in charge of stimulating mitochondrial outer membrane permeabilization. Studies have shown that the interconnection of BH3-only proteins elevates the release of BAK or BAX [60].

3) Those that control and regulate BCL2 proteins comprise PUMA, NOXA, BIK, HRX, BAD, BIM, BID, and BMF [50]. Reactions to different stress signals are controlled by the third category of the BCL2 family of proteins [56]. Recent findings have discovered that a correlation can be found between the BID and BID. The findings suggest that the BID can be triggered by death signals transmitted through the Fas/TNF-R1 death receptors. The singals are then transmitted and transmit these signals to the mitochondria through its cleaved product, truncated BID (tBID). Actually, the activation of caspase 8 leads to the cleavage of BID. This process is a critical step in the Fas pathway of apoptosis, where tBID translocates to the mitochondria and triggers apoptotic signals. The cleavage of BID by caspase 8 occurs within a native complex on the mitochondrial membrane, and the resulting tBID is involved in the activation of the mitochondrial apoptotic pathway. These findings shed light on the molecular mechanisms underlying apoptotic signaling through the Fas/TNF-R1 death receptors and the pivotal role of BID in this process [61,62]. It is noteworthy that BCL2 proteins are essential for p53-mediated apoptosis. Moreover, *Puma/Bbc3* and *Noxa/Pmaip* are induced by p53 [63]. In response to several intracellular and extracellular stress, such as hypoxia and DNA damage, a set of genes that participate in energy metabolism, cell-cycle arrest, or apoptosis are activated by p53, a key element in tumor suppression [64]. P53 can also stimulate autophagy, which aids in the suppression of tumors. Furthermore, P53 modulates numerous metabolic pathways for the metabolism of glucose, lipids, and amino acids. Thus, it aids in the cell's potential to resist and adapt to modest metabolic stress [65]. The mutated form of p53 can be found in more than half of human tumors, and it has been shown that inactivation of the p53 pathway is achieved by MDM2 and MDM4 upregulation [64]. For instance, in an *in-vitro* experiment, after cloning the MDM2 gene in the BALB/c 3T3 cell line (developed from disaggregated BALB/c mouse embryos, which are widely used in cancer-related research), it was observed that the overexpression of the MDM2 gene increases the tumorigenic ability of the cells [66]. At first, the expression of the MDM2 gene is regulated by the binding of p53 to the promoter. As the level of MDM2 rises, the p53 is inactivated by attaching and districting the transactivation domain [67]. RG7388 (idasanutlin) inhibits the formation of the p53-MDM2 complex and ultimately induces apoptosis, which exerts its function depending on the phase of the cell cycle [68]. Also, it can have an influential anti-AML role (especially in combination with venetoclax). MDM4 has been identified as an MDM2 homolog; both are identical in their p53-binding domain and essentially inhibit the role of p53. Therefore, p53 is one of the key regulators and controllers of apoptosis and a target for suppressing tumors [69]. Active clinical trials that are aimed to inhibit MDM-2 are summarized in Table 1.

**Table 1:** Summary of the clinical trials of the drugs that inhibit MDM2.

Drug	Phase	Status (Result)	Sponsor	Number of participants	Reference or Clinicaltrials.gov identifier
RG7112	1	Completed	Hoffmann-La Roche	116	NCT00623870
Idasanutlin	1/2	Terminated	Hoffmann-La Roche	24	NCT03850535
Idasanutlin	3	Terminated	Hoffmann-La Roche	447	NCT02545283
Idasanutlin	1	Completed	Hoffmann-La Roche	88	NCT02670044
Idasanutlin	1/2	Recruiting	Hoffmann-La Roche	220	NCT04029688
AMG-232	1	Recruiting	National Cancer Institute (NCI)	34	NCT04190550
APG-115	1	Recruiting	Ascentage Pharma Group Inc.	90	NCT04275518
Milademetan	1	Completed	Daiichi Sankyo Co., Ltd.	14	NCT03671564
Milademetan	1	Recruiting	Daiichi Sankyo, Inc.	156	NCT03552029
Milademetan	1/2	Recruiting	M.D. Anderson Cancer Center	58	NCT03634228
Milademetan	1	Active, not recruiting	Daiichi Sankyo, Inc.	200	NCT02319369

### 3.3 BCL2 family inhibitors pathways and drugs

As shown in Fig. 2, the BCL2 inhibitors include oblimersen, obatoclax mesylate (GX15-070), ABT-737, ABT-263 (navitoclax), ABT-199 (venetoclax), and S63845 [59]. These drugs inhibit BCL2 and activate the intrinsic apoptosis pathway.

A phosphorothioate antisense oligonucleotide, called oblimersen, is directed at the bcl-2 mRNA. The first six codons of the human BCL2 mRNA are targeted by oblimersen, reducing the expression level of BCL2 and ultimately increasing cell apoptosis [70].

Obatoclax mesylate, the first BH3 mimetic that has been used in clinical trials, applies its effectiveness by binding and interacting with the BH3-binding site of category 1 of the BCL2 family of proteins. Obatoclax is a BCL2 antagonist that can increase cytochrome C's release from mitochondria and reduce cell viability in AML [71]. It can cause a complete and rapid liberation of BAK from MCL1 and therefore helps overcome and regulate the MCL1-mediated resistance to apoptosis [72].

ABT-737 is an inhibitor of the BCL2 family of proteins, including BCL2L1, BclW, and BCL2 proteins, which induces apoptosis by death signals [73]. As ABT-737 binds to MCL1, ABT-737 resistance can be due to the overexpression of MCL1, which decreases the sensitivity of the drug [74]. In addition, it is worth mentioning that the cellular cytotoxic function of ABT-737 needs the expression of either BAK or BAX. On account of these reports, it can be resulted that a regulated level of the BCL2 family of proteins is required for the proper function of ABT-737 [75].

One of the restrictions of ABT-737 is that it cannot be used orally. However, this limitation has been overcome by discovering navitoclax. It has been discovered that navitoclax can inhibit tumor progression by inhibiting BCL2. Yet, because of the BCL-XL inhibition effect of Navitoclax, thrombocytopenia has been reported [76]. Furthermore, a functional synergism between 5-azacytidine (5-Aza) and ABT-737 in myeloid malignancies has been reported [77].

Venetoclax is also a BH3 mimetic, which selectively inhibits BCL2 and BCLW, and unlike ABT-737, it can be administrated orally [60]. No difficulties in the circulation of platelets and thrombocytopenia for ventocalx were recorded as it cannot inhibit BCL2L1 [59]. Several factors are reported to play role in developing resistance to Venetoclax, including but not limited to the mitochondrial protein Optic Atrophy 1, nicotinamide phosphoribosyltransferase, MCL1, alterations in the mitochondrial respiration and oxidative phosphorylation due to mitochondrial caseinolytic protease P activity and even phenotypical features like monocytic subclone [[78], [79], [80], [81]]. For instance, the overexpression of MCL1 suppresses the expression of Bim and induces an innate venetoclax resistance mechanism [82]. To solve this issue, venetoclax has been used in combination with cytarabine or daunorubicin, which ultimately decreases the MCL1 level [83]. From all of the BCL2 inhibitors, the combination of venetoclax with azacitidine or decitabine has obtained FDA approval to be used for patients more than 65 years old. This new drug combination could have promising effects compared to the standard induction chemotherapy in the mentioned age group [84].

Studies have revealed that S63845 exhibits a pronounced potency as an MCL1 inhibitor, demonstrating a more robust impact on MCL1 when compared to other inhibitors in its class, such as venetoclax and navitoclax. This distinction underscores the potential of S63845 as a notably effective agent in targeting and inhibiting the MCL1 protein, a critical component in the regulation of cell death and survival [85]. However, it has been indicated that the combination of navitoclax and S63845 is toxic, as their combination would induce apoptosis in platelets. Studies have shown that their combination is also toxic for several stem cells, causing tissue repair impossible [86].

Several other combination therapies have also been studied, mainly in resistant AML models [87]. Alvocidib, isolated from rohitukine (a derivate from a plant endemic to India), is an example in this regard. In principle, it is a semi-synthetic flavonoid, which is also known as NSC649890, flavopiridol, and L868275 [88]. Yet, it has been discovered that a combination of venetoclax and alvocidib cannot directly decrease MCL1. Nonetheless, it significantly increases NOXA, PUMA, BIM, and NBK [87].

Several studies have been conducted on a combination of P13K (an intracellular signaling pathway in which its activation has been detected in almost 50 % of AML samples) inhibitors such as taselib or GOC-0980 and venetoclax, particularly in resistant cases. It has been shown that they induce BAK and BAX activation and may result in apoptosis. Therefore, it can be considered that this combination has a decisive anti-AML role [89]. It has also been documented that the venetoclax and 5-Aza compounds can be used in myeloid malignancies. In theory, 5-Aza substantially reduces the MCL1 level [90]. Table 2 summarizes active clinical trials that are aimed to develop the Bcl-2 family of protein inhibitors.

**Table 2:** Summary of the clinical trials of the drugs that inhibit the BCL2 family of proteins.

Drug	Mechanism of action	Combination with	Related clinical trial	Number of participants	phase	Reference(s) or Clinicaltrials.gov identifier
Oblimersen	BCL2 antisense oligonucleotide	Gemtuzumab Ozogamicin	Oblimersen and Gemtuzumab Ozogamicin in Treating Older Patients with Relapsed Acute Myeloid Leukemia	N/A	2	NCT00017589
Obatoclax mesylate	BH3 mimetic Binding to the BH3-binding site of BCL2, BCL2L1, BCL-W, BCL-B, MCL1, and A1	Vincristine Sulfate, Doxorubicin Hydrochloride, and Dexrazoxane Hydrochloride	Obatoclax Mesylate, Vincristine Sulfate, Doxorubicin Hydrochloride, and Dexrazoxane Hydrochloride in Treating Young Patients with Relapsed or Refractory Solid Tumors, Lymphoma, or Leukemia	22	1	NCT00933985
Obatoclax mesylate	BH3 mimetic Binding to the BH3-binding site of BCL2, BCL2L1, BCL-W, BCL-B, MCL1, and A1	_____	Study of Obatoclax in Previously Untreated Acute Myeloid Leukemia (AML)	18	2	NCT00684918
Obatoclax mesylate	BH3 mimetic Binding to the BH3-binding site of BCL2, BCL2L1, BCL-W, BCL-B, MCL1, and A1	_____	Obatoclax Mesylate in Samples from Young Patients with Acute Myeloid Leukemia	50	N/A	NCT01150656
Obatoclax mesylate	BH3 mimetic Binding to the BH3-binding site of BCL2, BCL2L1, BCL-W, BCL-B, MCL1, and A1	_____	Safety and Efficacy of Obatoclax Mesylate (GX15-070MS) for the	44	1	NCT00438178
Venetoclax	BH3 mimetic Inhibiting BCL2 and BCL-W	Cytarabine	A Study of Venetoclax in Combination with Low Dose Cytarabine Versus Low Dose Cytarabine Alone in Treatment-Naive Patients with Acute Myeloid Leukemia Who Are Ineligible for Intensive Chemotherapy	211	3	NCT03069352
Venetoclax	BH3 mimetic Inhibiting BCL2 and BCL-W	Cytarabine	A Study Evaluating Venetoclax in Combination with Low-Dose Cytarabine in Treatment-Naïve Participants with Acute Myelogenous Leukemia	94	2	NCT02287233
Venetoclax	BH3 mimetic Inhibiting BCL2 and BCL-W	Cladribine, Idarubicin, Cytarabine	Cladribine, Idarubicin, Cytarabine, and Venetoclax in Treating Patients with Acute Myeloid Leukemia, High-Risk Myelodysplastic Syndrome, or Blastic Phase Chronic Myeloid Leukemia	408	2	NCT03586609
Venetoclax	BH3 mimetic Inhibiting BCL2 and BCL-W	Azacitidine, Decitabine	Study of ABT-199 (GDC-0199) in Combination with Azacitidine or Decitabine (Chemo Combo) in Subjects with Acute Myelogenous Leukemia (AML)	52	2	NCT05362942
Venetoclax	BH3 mimetic Inhibiting BCL2 and BCL-W	_____	A Study to Describe the Safety and Effectiveness of Venetoclax in Acute Myeloid Leukemia (AML) Patients (REVIVE Study) (REVIVE)	100	N/A	NCT03987958
Venetoclax	BH3 mimetic Inhibiting BCL2 and BCL-W	_____	A Study of the Effectiveness of Venetoclax Tablets in Adult Acute Myeloid Leukemia Participants Ineligible for Standard Induction Therapy in Russian Federation (INNOVATE)	50	N/A	NCT04253314
Venetoclax	BH3 mimetic Inhibiting BCL2 and BCL-W	_____	Venetoclax Registry (VENreg)	100	N/A	NCT03662724
Venetoclax	BH3 mimetic Inhibiting BCL2 and BCL-W	_____	A Phase 2 Study of ABT-199 in Subjects with Acute Myelogenous Leukemia (AML)	32	N/A	NCT01994837
Venetoclax	BH3 mimetic Inhibiting BCL2 and BCL-W	Azacitidine Rituximab/IDEC-C2B8	Study Evaluating Venetoclax in Subjects with Hematological Malignancies	38	1/2	NCT02265731
Venetoclax	BH3 mimetic Inhibiting BCL2 and BCL-W	_____	An Extension Study of Venetoclax for Subjects Who Have Completed a Prior Venetoclax Clinical Trial	550	3	NCT03844048
Venetoclax	BH3 mimetic Inhibiting BCL2 and BCL-W	_____	Expanded Access to Venetoclax	N/A	N/A	NCT03123029
AZD5991	Selective MCL1 inhibitor	Venetoclax	Study of AZD5991 in Relapsed or Refractory Haematologic Malignancies.	70	1	NCT03218683
Flavopiridol	Inhibiting MCL1 transcription	Cytarabine, Daunorubicin	Ph I Study of Alvocidib and Cytarabine/Daunorubicin (7 + 3) in Patients with Newly Diagnosed Acute Myeloid Leukemia (AML).	32	1	NCT03298984
Flavopiridol	Inhibiting MCL1 transcription	mitoxantrone hydrochloride, Cytarabine	Alvocidib, Cytarabine, and Mitoxantrone in Treating Patients with Newly Diagnosed Acute Myeloid Leukemia	45	2	NCT00407966
Flavopiridol	Inhibiting MCL1 transcription	mitoxantrone hydrochloride, Cytarabine, Daunorubicin	Alvocidib, Cytarabine, and Mitoxantrone Hydrochloride or Cytarabine and Daunorubicin Hydrochloride in Treating Patients with Newly Diagnosed Acute Myeloid Leukemia	172	2	NCT01349972
Flavopiridol	Inhibiting MCL1 transcription	mitoxantrone hydrochloride, Cytarabine	Flavopiridol, Cytarabine, and Mitoxantrone in Treating Patients with Relapsed or Refractory Acute Leukemia	35	1	NCT00470197
Voruciclib	Inhibiting MCL1 transcription	_____	A Phase 1 Study of Voruciclib in Subjects With B-Cell Malignancies or AML	92	1	NCT03547115
BEZ235	Inhibiting MCL1 translocation	_____	A Phase I, Dose-finding Study of BEZ235 in Adult Patients with Relapsed	23	1	NCT01756118
S64315	MCL1 inhibitor	Azacitidine	Phase I/II Trial of S64315 Plus Azacitidine in Acute Myeloid Leukemia	180	1/2	NCT04629443
S64315	MCL1 inhibitor	Venetoclax	Phase I Dose Escalation Study of Intravenously Administered S64315 in Combination with Orally Administered Venetoclax in Patients with Acute Myeloid Leukemia.	40	1	NCT03672695
S64315	MCL1 inhibitor	____	Phase I Study of S64315 Administered Intravenously in Patients with Acute Myeloid Leukemia or Myelodysplastic Syndrome	38	1	NCT02979366
Sorafenib	Inhibiting MCL1 translocation	Selinexor	Phase I/II, Study of Selective Inhibitor of Nuclear Export (SINE) Selinexor (KPT-330) + Sorafenib in Acute Myeloid Leukemia	17	2	NCT02530476
Sorafenib	Inhibiting MCL1 translocation	Asparaginase, Cytarabine, Bortezomib, Daunorubicin Hydrochloride, Etoposide, Mitoxantrone Hydrochloride	Bortezomib and Sorafenib Tosylate in Treating Patients with Newly Diagnosed Acute Myeloid Leukemia	1645	3	NCT01371981
Sorafenib	Inhibiting MCL1 translocation	Azacitidine	Sorafenib Plus 5-Azacitidine Initial Therapy of Patients with Acute Myeloid Leukemia (AML) and High-Risk Myelodysplastic	16	2	NCT02196857
Sorafenib	Inhibiting MCL1 translocation	Cytarabine	Sorafenib and Low Dose Cytarabine in Older Patients with Acute Myeloid Leukemia or High-Risk Myelodysplastic Syndrome	21	2	NCT00516828
Sorafenib	Inhibiting MCL1 translocation	Azacitidine	Sorafenib and 5-Azacitidine in Acute leukemia + Myelodysplastic Syndrome	60	2	NCT01254890
Sorafenib	Inhibiting MCL1 translocation	Azacitidine Cytarabine, Daunorubicin Hydrochloride	Sorafenib Tosylate and Chemotherapy in Treating Older Patients with Acute Myeloid Leukemia	54	2	NCT01253070

## 4 Death receptor pathways

Death receptor pathways are activated by tumor necrosis factor (TNF), CD95 (Apo1, fas), and TNF-related apoptosis-inducing ligand (TRAIL) receptors [91]. Three similar proteins are suggested to be the main receptors of TRAIL: TRAILR1, TRAILR2, and TAILR3 [92]. It has been reported that dysregulated expression of TRAILR3 can lead to apoptosis resistance [91]. TRAIL receptors are indeed important for inducing cell apoptosis; TRAILR2, TRAILR1, and fas bind to their intrinsic ligands and form the death-inducing signaling complex (DISC). Ultimately, DISC induces caspase-8 recruitment and initiates cell apoptosis [92]. In addition to the previously mentioned receptors, there is the Fas-associated protein with death domain (FADD). FADD acts as an intermediary between death receptor signaling and the caspase cascade. It is essential for the initiation of extrinsic apoptotic cell death [93].

It has been discovered that the c-Flip factor has a vital role in inhibiting death receptor signaling by restraining caspase-8 recruitment and DISC formation Practically, because of the direct and indirect function of caspase-9, c-Flip plays a crucial role in blocking apoptosis (e.g., by affecting caspase-5 or beginning the intrinsic pathway of apoptosis in a direct pathway) [91].

A human monoclonal antibody (HGS-ETR1; mapatumumab) has been used for targeting TRAILR1 [94]. In theory, both proapoptotic pathways (the intrinsic pathway and the extrinsic pathway) can be triggered by mapatumumab [91]. Moreover, it causes TRAILR1 activation and consequently triggers a caspase cascade, eventually leading to apoptosis. In addition to HGS-ETR1, HGS-ETR2 has been detected for targeting TRAILR2 and potentially can be used in combination with either paclitaxel or carboplatin [94].

## 5 Role of inhibitor of apoptosis proteins in AML treatment

The IAP family is an antiapoptotic protein that plays a critical role in controlling both extrinsic and intrinsic apoptosis pathways by binding to caspases [24]. In general, eight IAP proteins have been discovered in humans, which are as follows: 1- X-linked inhibitor of apoptosis (XIAP), 2- cellular IAP (cIAP1 or BIRC2), 3- cIAP2 or BIRC3, 4- surviving (BIRC5), 5- MLIAP (BIRC7), 6- BIRC6, 7- IAP-like protein (ILP2 or BIRC8), and 8- neuronal apoptosis inhibitory protein (BIRC1) [95]. Table 3 summarizes drugs that inhibit antiapoptotic pathways.

**Table 3:** Summary of the drugs inhibiting antiapoptotic pathways.

Drug	Mechanism of action	Route of administration	Common side effects	Reference or clinicaltrials.gov identifier
Idasanutlin	inhibiting the formation of the P-53-MDM2 complex	IV	Diarrhea, loss of appetite, bleeding problems	NCT02670044
				NCT04029688
Milademetan	Inhibits MDM-2	orally	Nausea, loss of appetite, platelet count decreased, fatigue, anemia	NCT03671564
				NCT03552029
Oblimersen	BCL2 antisense oligonucleotide	Continuous IV infusion	Nausea, thrombocytopenia, pyrexia, fatigue, anemia, vomiting	NCT00085124
Obatoclax mesylate	BH3 mimetic Binding to the BH3-binding site of BCL2, BCL2L1, BCL-W, BCL-B, MCL1, and A1	IV infusion	Neutropenia, thrombocytopenia, anemia, bleeding, fatigue	NCT00684918
				NCT01150656
				NCT00438178
Venetoclax (FDA approved)	BH3 mimetic Inhibiting BCL2 and BCL-W	orally	Nausea, diarrhea, anemia, upper respiratory infection, thrombocytopenia, fatigue	NCT03987958
				NCT02265731
				NCT03844048
				NCT03123029
S64315	MCL1 inhibitor	IV infusion	Tumor lysis syndrome, heart injury, fever	NCT03672695
Sorafenib	Inhibiting MCL1 translocation	orally	Bleeding gums, blood in urine or stools, coughing blood, redness of the hands, difficulty with breathing	NCT00516828

Practically, XIAP, CIAP, and MLIAP bind to caspases 3, 7, and 9 through their BIRs (baculovirus inhibitors of apoptosis) [96]. One to three copies of the BIR domain have been detected in each IAP protein. It has been well-recognized that these BIR domains of IAP proteins facilitate their binding to the caspases or proteins that organize apoptosis, which leads to the inhibition of targeted proteins. It has been shown that all IAP proteins have at least one BIR domain, which is in charge of their attachment to the caspases [97]. As mentioned above, some IAP proteins, such as XIAP, may have three BIR domains (BIR 1–3). These domains do not function similarly. The BIR1 domain of XIAP induces NfκB and TAK1 activation by particularly interfacing with Table 1. BIR2 targets preactivated caspase-3 or -7, while BIR3 was found to inhibit the caspase-9 activity. It has been shown that only a single BIR domain is adequate for their function, including cell survival [95]. TRAF1-TRAF2 heterocomplex is required in cIAP1 and cIAP2 recruitment in the TNRF2 (death receptor) signaling [98]. Practically, cIAP2 and cIAP1 participate with TRAFs in the TNF signaling pathway and, ultimately, regulate and facilitate the activation of MAP kinase in addition to the TNF-mediated NF-κB [99].

Smac20 (DIABLO21) has been identified as another significant regulator of apoptosis. It is released in parallel with cytochrome C from mitochondria into the cytosol and, eventually, inhibits IAPs [100]. Besides that, another IAP inhibitor, named embelin, inhibits XIAP by binding to BIR2 and BIR3 domains. It is worth mentioning that AML cell viability reduction is obtained from the combination of embelin and venetoclax [101]. Fig. 3 depicts how available drugs like Ventoclax, Idasanutlin, Mapatumumab, and Embelin can activate caspases.

**Fig. 3:** This figure illustrates the intrinsic and extrinsic pathways of apoptosis, highlighting the roles of the central regulators such as Bcl-2 and MCL-1 in the intrinsic pathway and the TRAIL receptor in the extrinsic pathway. Therapeutic agents like Venetoclax inhibit Bcl-2, Idasanutlin targets the intrinsic pathway, Mapatumumab activates TRAIL receptors, and Embelin and Smac20 (DIABLO21) reduce IAPs. These interactions ultimately activate the caspases, the main mediators of apoptotic cell death.

## 6 Conclusion

In AML treatment, the initiation of pharmacology and biotechnology has introduced targeted therapeutics addressing specific cancer cell pathways. Despite this progress, challenges like chemoresistance, relapse, and severe side effects persist. A deeper insight into the molecular mechanisms of AML's onset, progression, and chemoresistance is crucial. Addressing chemoresistance, a common obstacle, involves strategic combinations of chemotherapeutic agents [102]. To fully combat chemoresistance, there's a need for novel chemotherapeutics, with current strategies focusing on targeted drug delivery, such as organ-specific, drug-loaded nanoparticles. These approaches aim to thwart resistance in AML cells and reduce adverse effects. Realizing these targeted therapeutics necessitates interdisciplinary collaboration, encompassing fields like medicine, pharmacology, biochemistry, genetics, and nanotechnology.

Regarding the molecular mechanisms involved in the incidence and relapse after CR, some of the key players here are the BCL2 family of proteins, IAPs, and MDM2 have been recognized as essential players at this point. Each of these antiapoptotic factors has admissible pathways, which eventually cause tumor development. Designing and developing drugs that aim to target these players can be a beneficial strategy to inhibit tumor development. The BCL2 inhibitors include ABT199 (venetoclax), ABT263 (navitoclax), oblimersen, ABT-737, obatoclax mesylate, and S63845. These drugs have confirmed mechanisms for inhibiting the BCL2 family of proteins. A fair number of clinical trials have been performed on them in different countries, yielding good results. Yet, only a summary of their clinical studies is given in Table 2. Besides the BCL2 inhibitors, the drug named RG7388 (idasanutlin) induces apoptosis by inhibiting the formation of the p53-MDM2 complex. It is worth mentioning that the combination of idasanutlin and venetoclax has shown an influential anti-AML function [69]. Still, more investigations are required to study the effect of idasanutlin in combination with other drugs to discover if their combination is rewarding in tackling both tumor growth and chemotherapy resistance. Each of these drugs can be considered a candidate for drug delivery and targeted therapy alone or in combination with other medications.

## 7 Challenges

### 7.1 Mimicking the tumor environment and side effects

Despite all these benefits and information from apoptosis and antiapoptotic factors, there are still challenges and problems in studies in this area. For instance, since the tumor is a three-dimensional (3D) structure and most observations have been produced in 2D cell culture systems, the obtained data from *in-*vitro studies with 2D cell cultures may not be able to mimic the exact mechanism of these drugs in the real tumor environment. For this reason, more studies on 3D cellular models need to be done, as 3D cell cultures provide similar tumor environments [103]. Moreover, ongoing clinical trials about the effectiveness of the drugs or their side effects must be completed in the future so that we can make the final decision regarding the use of the drug. Another issue that must be considered when analyzing the results acquired from clinical trials is to evaluate the efficacy of chemotherapeutic agents on different classifications of AML or different stages of this disease.

In the coming years, more studies on apoptosis mechanisms and antiapoptotic factors will be performed. Indeed, more results will be published from the studies on the mentioned drugs. In the next few, distinctively, research will be focused on the elimination of the side effects of these drugs, enhancements in their efficacy, and availability. More studies will be conducted based on the idea of targeting cancer cells and delivering chemotherapeutic agents to the cancer cells/tissue specifically. It can be assumed that in the near future, a variety of drugs that are designed to aim these pathways will be approved by food and drug associations across the world. However, we expect that drugs with fewer side effects will be designed and undergo clinical trials with great hope of treating AML.

### 7.2 Relapce in AML

Despite recent approaches in the field of AML treatment, the side effects of medications or relapse of this disease have not reached their minimum, so clinical trials must aim to reduce risks and optimize the recovery of patients. As mentioned in this paper, targeting the BCL2 family, IAP, and death receptor proteins are novel approaches that can be used in AML treatment. Regarding BCL2 proteins, venetoclax is a novel BCL2 inhibitor which resolved some of the complications of previous BCL2 inhibitors, like having no difficulties in the circulation of the platelets and thrombocytopenia. It can be used orally in combination with other drugs for treating AML or resistance forms of that. Also, it is worth mentioning that venetoclax has been approved in Europe and the US for the treatment of AML patients who are inappropriate for severe chemotherapy. Ultimately, we suggest further experiments in this area to achieve reliable results. For this purpose, well-designed clinical trials that consist of a statistically significant number of patients are required. Additionally, an important topic that was not discussed in this paper is clonal evolution and its association with relapse and resistance. One recent perception is the existence of mechanism of resistance to a drug in some subclones. The selection killing of the AML bulk cells gives an opportunity for the pre-existing resistant clone to expand, leading to drug resistance. Also, more narrative reviews and/or systematic ones are needed to present new findings in treating AML by focusing on one of the current treatment options and its mechanism of action.

## CRediT authorship contribution statement

**Zahra Koolivand:** Writing – original draft. **Farbod Bahreini:** Writing – review & editing. **Elham Rayzan:** Writing – review & editing, Supervision. **Nima Rezaei:** Writing – review & editing, Supervision.

## Ethics approval and consent to participate

This article does not contain any studies with human participants or animals performed by any of the authors.

## Data availability statement

No data was used for the research described in the article.

## Funding

The authors did not receive any financial support for this article.

## Declaration of competing interest

The authors declare that they have no known competing financial interests or personal relationships that could have appeared to influence the work reported in this paper.
